# Practice and Discussion on the Management Mode of Comprehensive Pharmacy under the Strategy of Healthy China

**DOI:** 10.1155/2022/5477995

**Published:** 2022-01-11

**Authors:** Jing Liao, Xiaoli Hua, Xuefeng Cai, Yuyong Su, Lixiu Yu

**Affiliations:** Department of Pharmacy, Union Hospital, Tongji Medical College, Huazhong University of Science and Technology, Wuhan 430022, China

## Abstract

**Objective:**

To explore the practice of comprehensive pharmacy management mode under the strategy of healthy China.

**Methods:**

Combining with hospital practice, the advantages and disadvantages of comprehensive pharmacy management mode were discussed and considered.

**Results:**

The comprehensive pharmacy has advantages in improving work efficiency, optimizing resource allocation, refining pharmacy management, checking the compatibility of Chinese and Western medicines, and improving service quality, and it also increases the labor intensity of staff and is prone to prescription dispensing errors.

**Conclusion:**

Hospitals with mature conditions and permission can use the management mode of comprehensive pharmacy.

## 1. Introduction

Hospital pharmacy is a branch of comprehensive applied pharmacy, which covers different departments. When setting up pharmaceutical departments, hospitals should conform to the concept of patient-centered. At the same time, it ensures the completion of prevention, medical treatment, and health care. At present, with the continuous reform of the medical system, the competitiveness of the pharmaceutical market is gradually increasing. All these urge the hospital pharmacy work to strengthen the transformation of work mode, so as to keep pace with the times. In recent years, the comprehensive pharmacy management mode has been adopted for pharmacy management, and good results have been achieved. Hospital pharmacy is a comprehensive department integrating management, technology, operation, and service. Its function is to accurately provide qualified drugs for patients, ensure their safe and effective use, and control medical expenses more economically and reasonably [1, 2]. With the rapid development of medical and health services, the competitiveness of the pharmaceutical market has also increased. In order for hospitals to adapt to the development of society, our daily management of pharmacies needs to keep pace with the times. Under the background of healthy China strategy, this paper discusses the practice of comprehensive pharmacy management mode.

## 2. Healthy China Strategy

The Fifth Plenary Session of the Eighteenth Central Committee of the Communist Party of China was put forward to promote the construction of a healthy China and upgrade “healthy China” into a national strategy. On this basis, the report of the 19th National Congress of the Communist Party of China further pointed out that “people's health is an important symbol of national prosperity and national prosperity” [3].

Implementing healthy China strategy is an urgent need for the development of the times and the common expectation of ordinary people. It is the party's solemn commitment to the people and a major popular project, and it is also an important manifestation of China's fulfillment of its international obligations and participation in global health governance. According to the report, by the second stage of this century, “people will enjoy a happier and healthier life.” The Chinese people will surely share the rich well-being of a healthy China and lay a healthy foundation for realizing the goal of “two centennials” and realizing the Chinese dream [4].

## 3. Management Mode of Comprehensive Pharmacy

Because the environment and conditions of each hospital are different, the Ministry of Health of China has no uniform regulations on the management of the pharmacy department of the hospital, and the pharmacy of each hospital can be built according to the actual situation. Comprehensive pharmacy is to set up a large pharmacy in the whole hospital, that is, to combine the outpatient pharmacy of traditional Chinese medicine, the outpatient pharmacy of western medicine and the inpatient pharmacy into one and manage all the pharmacy works in the hospital. The staff of the general pharmacy is concentrated, which is convenient for the daily work of the hospital and suitable for the actual situation of the hospital. To integrate the staff of the general pharmacy in our hospital and manage drugs reasonably, pay attention to the following points:

### 3.1. Hospital System Construction

Pharmacy staff should have the idea of serving the majority of patients wholeheartedly and noble drug ethics, be serious and responsible for their work, control the quality of drugs, and ensure the safety and effectiveness of patients' medication. Medical institutions shall distribute drugs in strict accordance with the requirements of diagnosis and treatment norms. The performance, usage, dosage, precautions, taboos, and other matters of the drug shall be explained when delivering the drug and false publicity shall not be made. The prescription reviewer shall not alter or substitute the drugs listed in the prescription. If there is any problem, he shall inform the prescription doctor and ask him to sign for confirmation or reissue the prescription. To realize the standardized management of pharmacy, it is necessary to formulate effective rules and regulations. In January 2019, under the guidance of hospital leaders, our department successfully merged outpatient western pharmacy, inpatient western pharmacy, and western medicine pharmacy into a comprehensive pharmacy, which realized centralized management of drugs and personnel, simplified pharmacy work flow, reduced error rate, and improved work efficiency and drug use turnover rate.

#### 3.1.1. Effect Evaluation

Observe the situation of drug matching and the satisfaction degree of clinical departments to pharmacy work before and after implementation and investigate all medical staff (especially nurses) with self-made satisfaction questionnaire of clinical departments and count the satisfaction of pharmacy work after the implementation of comprehensive pharmacy management mode, including satisfaction, better satisfaction, general satisfaction, and dissatisfaction, with satisfaction + better satisfaction/total number; 90–100 points: highly recognized and satisfied with the pharmacy work; 80–89 points: satisfied with the pharmacy work and can get the required drugs quickly and accurately every day; 70–79 points: the pharmacy work needs to be improved and generally satisfied; below 69 points: the work efficiency of pharmacy staff is not improved or the work of medical staff is disturbed and dissatisfied.

Comparison of satisfaction of medical staff before and after management: the satisfaction of medical staff before and after management is 82.14%, 96.43%, and the satisfaction of medical staff after management is obviously higher than that before management, as shown in Table 1.

In order to ensure the effective implementation of the rules and regulations, we require all the staff of medicines and pharmacies in the hospital to be included in the management scope of pharmacy department and implement the post responsibility system, which is fully responsible by the Pharmacy Management Committee, and clarify the post responsibilities of pharmacy department director, pharmacy team leader, storekeeper, buyer, and drug dispenser. Strengthen personnel management: it should have good professional ethics, and it is strictly forbidden to abuse drugs or take drug rebates. Hospitals regularly educate and train pharmaceutical personnel on medical ethics; standardize the service language; patiently, carefully, and professionally answer patients' drug consultation; improve the ability to communicate with others; and establish a good professional image. Detailed medication precautions to patients to ensure medication safety and making the original passive provision of drugs become active provision of pharmaceutical services are also conducive to collecting information on adverse reactions of drugs. Drug quality management is the top priority to prevent drug accidents. The acceptance of drugs from the drug warehouse to the pharmacy shall be carried out quickly, and the variety, specification, number of phases, and packaging shall be considered, so as to avoid failure and waste in the rabbit phase as far as possible. The staff of the pharmacy shall check the prescription and avoid the supply of expired drugs to patients [5, 6]. Actively accept the supervision of the masses, improve work efficiency, reduce deployment errors, change the image of the window, and improve the quality of pharmaceutical care.

### 3.2. From Preventing and Treating Diseases to Maintaining and Promoting Health

Traditional Chinese medicine in the comprehensive pharmacy management mode is a typical personalized and continuous health management and service mode, which is comprehensive in terms of influencing factors, from public policy to production and living environment, from medical and health services to lifestyle and genetic factors [7]. The whole cycle runs through a person's life, from the beginning of pregnancy, to pregnancy, fetus, infant and childhood, adolescence, adulthood, and finally to old age. The role of Chinese medicine is to integrate health into all policies and establish a health impact assessment system.

### 3.3. Centralized Management of Drugs and Personnel, Detailed Pharmacy Work, Clear Job Responsibilities to Individuals

The management and storage of drugs in general pharmacies are concentrated in the same area, and corresponding personnel are set up to manage drugs on special shelves, register the records of drugs in near term period, and register the records of drugs off shelves and expired drugs to ensure that all drugs used are within the validity period.

According to the statistics of related projects in January 2019 after the implementation of comprehensive pharmacy management in outpatient pharmacies, compared with before the implementation (December 2019), the error rate of dispensing, invalid drugs, and waiting time for taking drugs in outpatient pharmacies decreased, and the satisfaction of patients with service improved. The results are shown in Table 2.

A special person is responsible for registering and adjusting the temperature and humidity of the general pharmacy. Prescription review, doctor's advice review, drug dispensing, drug application and storage, prescription management, etc., all have special personnel in charge, and all kinds of personnel have clear work and responsibilities, which accurately refines the work of the comprehensive pharmacy as a whole, so that the work of the comprehensive pharmacy can be carried out smoothly and orderly. In addition, all staff in the department implement unified scheduling, flexibly arrange pharmacy work, and facilitate post adjustment.

### 3.4. Make Full Use of Informatization

With the vigorous development of medical information technology, digital office has been basically realized in general hospitals at all levels. In the future, multimedia devices such as computers and handheld computers will run through the business processes of various departments in hospitals such as hospital management system (HIS) and rapid dispensing system (EDS). The former can reduce drug pricing, charging and taking time and ensure accurate and uniform prices by simplifying pharmacy charging procedures, thus avoiding medical disputes; The latter directly realizes the information management of computer data input and transmission. Under the mode of process diversion and division of labor and cooperation, drugs are reassembled after bar code scanning, which is convenient for pharmacists to check and provide efficiency and accuracy.

### 3.5. Economical and Rational Drug Use

Comparison of drug qualification before and after management: the drug qualification rate in pharmacy before management is 85%, and after management is as high as 95%, which is obviously higher than that before management, as shown in Table 3.

The original oral medicines are imported into the system in the smallest package. Considering that some medicines are packed in too many packages and the price is relatively high, the medicines are imported into the system in the smallest unit after the establishment of the comprehensive pharmacy, so as to avoid the drug abuse phenomenon caused by the overtreatment of prescriptions prescribed by doctors and at the same time reduce the economic burden of patients, thus realizing the principle of safe, effective, and economical rational drug use.

## 4. Some Disadvantages of Comprehensive Pharmacy

### 4.1. Expand the Medicine Dispensing Refusal and Increase the Labor Intensity of the Staff

After the implementation of comprehensive pharmacy management, western medicines and Chinese patent medicines should be placed in one window at the same time, especially the large volume of most Chinese patent medicines, which makes the medicine cabinet in the window multiply. After the expansion of space, the dispensing distance becomes longer, which increases the labor intensity of drug dispensing personnel and then easily leads to drug dispensing errors [8].

### 4.2. There Are Many Batch Numbers in Drug Inventory, Which Are Easy to Be Confused

After the establishment of a comprehensive pharmacy, different batch numbers of drugs are easy to be placed in disorder. If the drug racks are not arranged in time, it is easy to mix different batch numbers of drugs, and drugs with long effective period are given priority over drugs with short effective period. In addition, scattered injection drugs are also prone to different batch numbers being put together.

### 4.3. If You Do Not Master the New Theory Thoroughly, It Is Easy to Make Prescription Dispensing Mistakes

First of all, in the trial prescription, the use of Chinese patent medicine pays attention to syndrome differentiation and treatment and increases and decreases with the symptoms. Without a certain theoretical basis of traditional Chinese medicine, the safety and effectiveness of Chinese patent medicine are often ignored. Similarly, the mastery of western medicine theory by Chinese medicine personnel is not comprehensive enough. Secondly, in the drug dispensing, especially in the initial stage of merger, the dispensing personnel's understanding of drugs only stays on some individual characteristics, but cannot comprehensively understand the composition and efficacy of drugs, which leads to some drugs with similar shapes, colors, or drug names being taken wrong and sent wrong [9].

### 4.4. There Are Hidden Dangers in the Security and Stability of Pharmacy Network System

At present, hospitals are all electronic prescriptions. Under the unified management mode of general pharmacies, the problems of slow network speed and system card should be taken into account. The information department should strengthen the compatibility of network systems and improve the system performance of computers.

## 5. Discussion

Hospital pharmacy is a branch of comprehensive applied pharmacy, which covers different departments. When setting up the pharmaceutical department, the hospital should comply with the concept of patient-centered. At the same time, ensure the completion of prevention, medical treatment, and health care. At present, with the continuous reform of the medical system, the competitiveness of the pharmaceutical market is gradually increasing. All these urge the hospital pharmacy work to strengthen the transformation of work mode, so as to keep pace with the times. In recent years, the comprehensive pharmacy management mode has been adopted for pharmacy management, and good results have been achieved. The research shows that the comprehensive management of hospital pharmacies reduces the allocation of pharmacy personnel, reduces the storage space and quantity of drugs, and simplifies the management process of drugs in pharmacies. Talent cultivation and construction is an important foundation to ensure the rapid development of various industries. The work function of pharmacy staff in the future development of hospital is not only to prescribe drugs but also to provide patients with various high value-added professional services such as medication consultation. Hospitals with conditions and needs can try this management mode, and colleges and universities can try to cultivate talents with Chinese and Western medicine to meet market demand. We should also pay attention to and try to solve some disadvantages exposed in practice.

In this study, it was found that 9 kinds of drugs were unqualified before management, and the qualified rate was 85%. Only 3 kinds of drugs were unqualified after management, and the qualified rate was as high as 95%. The qualified rate of drugs in pharmacies after management was significantly higher than that before management (*P* < 0.05). The satisfaction of clinical departments before and after management was 82.14% and 96.43%, respectively. The satisfaction of medical staff after management was significantly higher than that before management (*P* < 0.05). The results showed that the comprehensive pharmacy management method could manage pharmacy drugs scientifically and effectively, avoid misplacement and expiration of drugs, and improve the work efficiency and clinical satisfaction of pharmaceutical staff, which was consistent with the current research.

One year's practice generally has more advantages than disadvantages, but there are still many problems that need to be improved and solved. Under the comprehensive pharmacy management mode, the professionalism of Chinese medicine practitioners is dispersed, the sense of mission is not stimulated, the sales volume of Chinese medicine declines, the maintenance quality of medicinal materials declines, the error rate of Chinese medicine allocation rises, and the social attention decreases, which makes the protection and development of Chinese medicine become more urgent. Under the background of healthy China, comprehensive pharmacy management also emphasizes giving priority to healthy development, financial funds should guarantee investment in health management, and public health resources should give priority to meeting health needs. At the same time, the health management of Chinese medicine should also implement supervision and accountability. People get health dividends.

## 6. Conclusion

The form of comprehensive pharmacy in our hospital is the successful application of business process reengineering in pharmacy care. Its advantages are obvious for both hospitals and patients, and its economic and social benefits are remarkable. Therefore, we should also conduct regular inspections on the comprehensive pharmacies established in hospitals, conduct comprehensive analysis in time once problems are found in the management process, and actively explore a scientific, reasonable, and sustainable development new model, so as to change the deficiencies existing in the model at that time. Under the strategy of healthy China, the pharmacy management in the future should continue to adhere to the system construction, promote information utilization, strengthen the management of traditional Chinese medicine preparations, attach importance to the construction of talent team, and carry out clinical pharmacy services in depth, so as to better reflect the hospital's patient-centered service concept and improve the hospital pharmacy service quality.

## Figures and Tables

**Table 1:** Compare satisfaction before and after management (*n* = 28).

Time	Satisfied	Quite satisfied	General satisfaction	Dissatisfied	Degree of satisfaction (%)
Before management	18	5	3	2	82.14
After management	20	7	1	0	96.43

**Table 2:** Comparison of related projects before and after the implementation of comprehensive pharmacy management.

Time	Adjustment error rate (%)	Waiting time for taking medicine (min)	Expired drugs (once/half a year)	Patient service satisfaction (%)
Before management	0.02	≤4	8	88.69
After management	0.01	≤2	4	92.37

**Table 3:** Drug eligibility in pharmacies before and after management (*n* = 60).

Time	Qualified	Disqualification	Percent of pass (%)
Before management	51	9	85
After management	57	3	95

## Data Availability

The data used to support the findings of this study are included within the article.
